# Circular RNA circ_0000467 regulates colorectal cancer development via miR-382-5p/EN2 axis

**DOI:** 10.1080/21655979.2021.1889130

**Published:** 2021-03-09

**Authors:** Lu Xie, Zhihong Pan

**Affiliations:** Department of Gastroenterology, The People's Hospital of China Three Gorges University and The First People's Hospital of Yichang, Yichang, Hubei Province, China

**Keywords:** circ_0000467, CRC, miR-382-5p, EN2

## Abstract

Circular RNAs (CircRNAs), belonging to non-coding RNAs, exert a crucial modulatory role in cancer progression. In this study, circRNA microarray analysis was utilized to screen differentially expressed circRNA in colorectal cancer (CRC) and circ_0000467 was identified as one circRNA whose expression was significantly upregulated in CRC. Quantitative reverse transcriptase-polymerase chain reaction (qRT-PCR) indicated that circ_0000467 and engrailed-2 (EN2) expression levels were up-modulated, while the expression level of miR-382-5p was down-modulated in CRC tissues. The depletion of circ_0000467 expression was found to impede the multiplication, migration, invasion, and epithelial-mesenchymal transition (EMT) processes in CRC cells, which were examined by 3-(4,5-dimethylthiazol-2-yl)-2, 5-diphenyltetrazolium bromide (MTT) and Transwell experiments. Dual-luciferase reporter assay was used to verify the targeting relationship between circ_0000467 and miR-382-5p. It was also revealed that circ_0000467 could up-regulate EN2 expression via repressing miR-382-5p in CRC cells. Furthermore, EN2 overexpression counteracted the suppressing effects of circ_0000467 knockdown on the malignant behaviors of CRC cells. To sum up, circ_0000467 facilitates CRC development by modulating the miR-382-5p/EN2 axis, and circ_0000467 is a promising target for CRC therapy.

## Introduction

Colorectal cancer (CRC) is the third most common carcinoma in China and poses a serious threat to people’s health [1]. About 25% of CRC patients suffer from distant metastases when they are diagnosed [2]. Tumor metastasis is a major cause of death in CRC patients [3]. Specifically, CRC patients with liver metastases only have a 5-year survival rate of 25–40%, even after the resection of the metastases [4]. Hence, probing the mechanisms of CRC progression and identifying novel targets are imperative.

Circular RNAs (CircRNAs) are circular non-coding (nc) RNA produced by covalently linking the 5' end and 3' end [5]. CircRNAs are stable and conserved, and they are usually expressed at specific developmental stages or in specific tissues [6]. CircRNAs are crucial in regulating different biological processes, for example, cell differentiation, multiplication, apoptosis and so on [7]. Emerging evidence implies that circRNAs are essential regulators in CRC progression [8,9]. Reportedly, circ_0026344 under-expression is linked to adverse prognosis in CRC patients [10]. Circ_0009361 is remarkably under-expressed in CRC, and the up-modulation of circ_0009361 expression enhances APC2 expression and restrains Wnt/β-catenin signaling, which impedes CRC development [11]. Moreover, circ_101555 is overexpressed in CRC, and circ_101555 knockdown suppresses cell multiplication, induces apoptosis, and impairs cellular DNA repair by modulating CDK6 and RPA3 [12]. Nevertheless, the roles and modulatory mechanisms of diverse circRNAs in CRC warrant further investigation. Circ_0000467 is a newly discovered circRNA, and it is a promising noninvasive biomarker for gastric cancer [13]. However, the exact role and mechanism of circ_0000467 in CRC progression is still obscure.

CircRNAs can modulate gene expression by working as competitive endogenous RNAs (ceRNAs) for microRNAs (miRNAs) [14]. MiRNAs are small ncRNAs with approximately 22 nucleotides in length and often work as tumor suppressors or oncogenes to modulate tumor progression [15]. For instance, miR-382-5p is under-expressed in CRC and associated with patients’ prognosis [16]. MiR-382-5p, reportedly, impedes the multiplication, migration, and invasion, and enhances chemosensitivity of CRC cells [17]. Nevertheless, the upstream regulatory mechanisms modulating the tumor-suppressive effects of miR-382-5p in CRC are undefined. Additionally, Engrailed-2 (EN2), is a homeobox-containing gene, and EN2 protein is an essential regulator during embryonic neural development, and normally, it is only expressed in Purkinje neurons and renal tubular epithelial cells [18]. Reportedly, EN2 expression is abnormally up-modulated in CRC and EN2 facilitates the multiplication and migration of CRC cells [19].

This work was aimed to identify whether circRNAs were aberrantly expressed in tissues of patients with CRC and to probe the biological function of circ_0000467 in CRC progression. The role of circ_0000467 and the molecular mechanism of circ_0000467/miR-382-5p/EN2 axis in CRC are explored, and it was demonstrated that circ_0000467 knockdown repressed the malignant biological behaviors of CRC cells via repressing miR-382-5p and up-regulating EN2.

## Material and methods

### CircRNA expression profile analysis

Two CRC microarray datasets (GSE138589 and GSE142837) were downloaded from the Gene Expression Omnibus (GEO) database and GEO2R online tool was employed to screen the differentially expressed circRNAs in CRC tissues (v.s. non-cancerous tissues).

### Tissue samples and cell lines

Tissue samples were available from subjects who had been diagnosed with CRC between 2015 and 2019 in the People’s Hospital of China Three Gorges University. Every participant enrolled in this work provided written informed consent and this study was endorsed by the Ethics Committee of the People’s Hospital of China Three Gorges University. Human colonic epithelial cell line (FHC) and CRC cell lines (SW480, SW620, HT29, RKO, and HCT116) were obtained from the American Type Culture Collection (ATCC, Manassas, VA, USA). Dulbecco’s Modified Eagle Medium (DMEM) (Thermo Fisher, Waltham, MA, USA) containing 10% fetal bovine serum (FBS, Gibco, Grand Island, NY, USA), 100 μg/mL streptomycin, and 100 U/mL penicillin (Invitrogen, Carlsbad, CA, USA) was utilized to culture the cells at 37°C with 5% CO_2_.

### Cell transfection

The CRC cells were transferred into a 6-well plate at 3 × 10^5^ cells/well. Small interfering RNA (siRNAs) targeting circ_0000467 (si-circ_0000467#1, si-circ_0000467#2, and si-circ_0000467#3), miR-382-5p mimics, pcDNA3.1-EN2, and their respective controls were from Biomics Biotech (Nanjing, China). Then, cell transfection was conducted by Lipofectamine 2000 (Thermo Fisher Scientific, Waltham, MA, USA) according to the manufacturer’s instruction.

### Quantitative real-time polymerase chain reaction (qRT-PCR)

Total RNA was isolated and quantified by TRIzol Reagent (Invitrogen, Carlsbad, CA, USA) and NanoDrop 2000 (Thermo Fisher Scientific Inc., Carlsbad, CA, USA). RNA was reversely transcribed into cDNA by ReverTra Ace qRT-PCR Kit (Toyobo, Osaka, Japan), and qRT-PCR was conducted with THUNDERBIRD SYBR qPCR Mix (Toyobo, Osaka, Japan). The gene expression was normalized by GAPDH/U6 expression. Relative quantification were performed using 2^−ΔΔCt^ method. The primers designed for this research were displayed in Table 1.

**Table 1.** Primer sequence

Gene	Sequence
circ_0000467	F: 5'- ACACAATGGGACTTAAAAATGCGA −3' R: 5'- ACAGATCATCTTTCACATCAGTCT −3’
EN2	F: 5'- CTACTGTACGCGCTACTCGG −3' R: 5'- CCCGTGGCCTTCTTGATCTT −3’
GAPDH	F: 5'- GGGAAATCGTGCGTGACATTAAG −3' R: 5'- TGTGTTGGCGTACAGGTCTTTG −3’
miR-382-5p	F: 5'- ATCCGTGAAGTTGTTCGTGG −3' R: 5'- TATGGTTGTAGAGGACTCCTTGAC −3’
U6	F: 5'- GCTTCGGCAGCACATATACTAAAAT −3' R: 5'- CGCTTCACGAATTTGCGTGTCAT −3’
Note: F, forward; R, reverse.	

### Subcellular RNA fractionation experiment

Cytoplasmic and nuclear RNA were extracted from CRC cells with NE-PER Nuclear and Cytoplasmic Extraction Reagents (Thermo Scientific, Waltham, MA, USA). Then, the RNA isolated from the nucleus or cytoplasm was analyzed with qRT-PCR. The expression levels of nucleus control (U6), cytoplasm control (GAPDH), and circ_0000674 were, respectively, measured.

### 3-(4, 5-dimethylthiazol-2-yl)-2, 5-diphenyltetrazolium bromide (MTT) assay

The cells were transferred into 96-well plates (3 × 10^3^ cells/well) and then incubated with 20 μL of MTT solution (5 mg/mL; Sigma, St. Louis, Mo, USA) for 4 h. Subsequently, 200 μL of DMSO (Sigma, St. Louis, Mo, USA) was supplemented, and the formazan was dissolved. Subsequently, a microplate reader was used to test the absorbance at 490 nm (Bio Tek Instruments, Inc., Winooski, VT, USA).

### Transwell experiment

The transfected cells (1 × 10^4^) were suspended in 200 μL of serum-free medium and planted into the top compartment of each Transwell insert (8 μM pore size, Costar, Shanghai, China). Medium containing 10% FBS was replenished to the lower compartment as the chemoattractant. The cells were cultured for 48 h for the invasion experiment and 24 h for the migration experiment. Next, the cells in the upper compartment were removed with cotton swabs, and the cells on the bottom surface were fixed with methanol and stained with 0.1% crystal violet. With three random areas of each Transwell insert, the number of migrated or invasive cells was counted under a microscope. Matrigel (BD Biosciences, San Jose, CA, USA) was used to cover the filter of the Transwell inserts for the invasion experiment, and it was not used in migration experiment.

### Dual-luciferase reporter gene experiment

The wild type (WT) circ_0000467/EN2 sequence containing the miR-382-5p binding site was amplified and inserted into the empty luciferase reporter vector to obtain the WT-circ_0000467/WT-EN2 reporter vector. The mutant type (MUT) circ_0000467/EN2 sequence was also inserted into the empty luciferase reporter vector to obtain the MUT-circ_0000467/MUT-EN2 reporter vector. The constructed luciferase reporter plasmids were co-transfected with miR-382-5p mimics or miR-control into HEK293T cells planted in a 96-well plate. After 48 h, the activities of Firefly luciferase and Renilla luciferase were determined using a dual-luciferase detection system (Promega, Madison, WI, USA). The relative luciferase activity was normalized to Renilla luciferase activity.

### RNA immunoprecipitation (RIP) experiment

The binding relationship between miR-382-5p and circ_0000467 was examined with Magna RIP Kit (EMD Millipore, Billerica, MA, USA). CRC cells were lysed in RIP buffer, and then incubated with magnetic beads conjugated with anti-AGO2 antibody or IgG for 4 h at room temperature. Next, the immunoprecipitate was treated with proteinase K to remove the protein, and then the RNA was isolated, and qRT-PCR was performed.

### RNA pull-down experiment

Pierce Magnetic RNA–Protein Pull-Down Kit (Thermo Fisher Scientific, Waltham, MA) was adopted for RNA pull-down experiment. The WT or MUT miR-382-5p sequence was synthesized and biotinylated. Then, Bio-miR-382-5p-WT/MUT was incubated with cell lysates overnight. Then, the pull-down mixture was collected for examining the relative enrichment of circ_0000467 using qRT-PCR.

### Western blot

Total proteins were extracted using radio immunoprecipitation (RIPA) lysis buffer (1% NP-40, 0.5% sodium deoxycholate, 50 mM Tris-HCl, 0.1% SDS, 150 mM NaCl, pH 7.5) containing 1% protease inhibitor. The protein sample (30 µg in each group) was separated by 10% SDS-PAGE and transferred onto the nitrocellulose membranes (Millipore, Bedford, MA, USA). After being blocked with 5% skimmed milk for 1 h at room temperature, the membranes were incubated with anti-GAPDH (Abcam, Cambridge, UK) (ab37168, 1:3000), anti-Vimentin (Abcam, Cambridge, UK) (ab8978, 1:3000), anti-E-cadherin (Abcam, Cambridge, UK) (ab40772, 1:3000), and anti-EN2 (ab45867, 1:500) primary antibodies (Abcam, Cambridge, UK) at 4°C for 12 h. Then, the membranes were incubated with a horseradish peroxidase-conjugated secondary antibody at 4°C for 2 h. Finally, the intensity of bands was analyzed using Image-Pro Plus 6.0 software (Media Cybernetics, Inc.) with Immobilon ECL substrate kit (Millipore, Billerica, MA, USA). GAPDH was utilized as an internal control.

### Statistical analysis

All statistical analyses were performed using SPSS version 19.0 software (SPSS, Inc, Chicago, IL, USA). Student’s *t*-test and one-way ANOVA were employed to perform the comparisons between the two groups and among multiple groups, respectively. A Chi-square test was applied for analyzing the correlation between circ_0000467 expression and clinicopathological characteristics. The linear correlation between circ_0000467-miR-382-5p and EN2-miR-382-5p expressions was analyzed by Pearson’s correlation analysis. *P* < 0.05 signified statistical significance.

## Results

### Circ_0000467 expression was up-modulated in CRC tissues

To probe into the expression characteristics of circRNAs in CRC tissues, microarray data of GSE138589 and GSE142837 downloaded from the GEO database were analyzed (log_2_|Fold change|>1.5, *P* < 0.05, Figure 1(a)). There were 43 up-modulated circRNAs in GSE138589 and 7 down-modulated circRNAs; in GSE142837, there were 20 differentially expressed circRNAs, including 5 circRNAs with up-modulated expression and 15 circRNAs with down-modulated expression (Figure 1(a)). Nonetheless, only hsa_cic_0000467 expression was significantly up-modulated in both GSE138589 and GSE142837 (Figure 1(b)). Additionally, qRT-PCR analysis unmasked that cic_0000467 expression was remarkably higher in 69 CRC tissues than in paracancerous tissues (Figure 1(c)). Meanwhile, by analyzing the association between clinicopathological features and cic_0000467 expression in 69 CRC patients, cic_0000467 overexpression was observed to be positively related to tumor size, histological grade, and TNM stage (Table 2). Subsequently, the data of qRT-PCR suggested that cic_0000467 expression was higher in human CRC cell lines than in FHC cell lines (Figure 1(d)). Besides, cic_0000467 was revealed to be predominantly localized in the cytoplasm by cellular RNA fractionation experiment (Figure 1(e)). These data implied that circ_0000467 might be a vital regulator in CRC progression via functioning as a ceRNA.

**Table 2.** Correlations between circ_0000467 expression and clinical characteristics in CRC patients

Pathological indicators	Number of patients	Circ_0000467		*P-value* (*P < 0.05)
		High expression	Low expression	
All cases	69	34	35	
Age				
<47	36	15	21	0.187
≥47	33	19	14	
Gender				
Female	21	12	9	0.387
Male	48	22	26	
TNM stage				
I–II	33	12	21	0.040*
III–IV	36	22	14	
Tumor size				
<5 cm	37	14	23	0.041*
≥5 cm	32	20	12	
Tumor location				
Colon	34	15	19	0.119
Rectum	35	22	13	
Histology grade				
Well	31	11	20	0.022*
Moderate/poor	38	24	14

**Figure 1.** The expression of circ_0000467 was up-modulated in CRC

a) Differential expression of circRNAs in GSE138589 and GSE142837. b) Circ_0000467 was dysregulated in both GSE138589 and GSE142837. c) Circ_0000467 expression in 69 paired CRC tissues and matched adjacent tissues was examined by qRT-PCR. d) Circ_0000467 expression in CRC cell lines (SW480, SW620, HT29, RKO, and HCT116) and the FHC cells was examined by qRT-PCR. e) The subcellular distribution of circ_0000467 was analyzed by cellular RNA fractionation assays. GAPDH was mainly localized in the cytoplasm and U6 was mainly localized in the nucleus, which were used as a negative control.***P < 0.001.

### Knockdown of circ_0000467 restrained the multiplication, migration, invasion, and epithelial-mesenchymal transition (EMT) process of CRC cells

Next, we studied the biological function of circ_0000467 in CRC cells. Based on the above data, circ_0000467 expression was relatively high in SW620 and HT29 cells, so three different siRNAs were transfected into SW620 and HT29 cells to construct a cell model with circ_0000467 under-expression. qRT-PCR data indicated circ_0000467 siRNA#1 had the strongest suppressing effects on circ_0000467 expression, so si-circ_0000467#1 (si-circ_0000467) was selected for the follow-up experiments (Figure 2(a)). MTT experiment illustrated that circ_0000467 knockdown markedly repressed the multiplication of both SW620 and HT29 cells (Figure 2(b)). Transwell experiment suggested that circ_0000467 knockdown also observably suppressed migration and invasion of CRC cells (Figure 2(c)). Western blot data revealed that E-cadherin protein expression was remarkably up-modulated and Vimentin was remarkably down-modulated after circ_0000467 knockdown (Figure 2(d)). The data indicated that circ_0000467 knockdown restrained the multiplication, migration, invasion, and EMT process of CRC cells.

**Figure 2.** Knockdown of circ_0000467 impeded the multiplication, migration, and invasion of CRC cells

a Three siRNAs against circ_0000467 (si-circ_0000467#1, si-circ_0000467#2, and si-circ_0000467#3) were transfected into SW620 and HT29 cells, and circ_0000467 expression was detected by qRT-PCR.b MTT experiment was performed to detect the multiplication of SW620 and HT29 cells after the transfection.c Transwell experiment was utilized to detect migration and invasion of SW620 and HT29 cells after the transfection.d Western blot was executed to detect the EMT markers in SW620 and HT29 cells after the transfection.*P < 0.05, **P < 0.01, and ***P < 0.001.

### Circ_0000467 sponged miR-382-5p in CRC cells

To probe into the underlying mechanism of circ_0000467 in CRC, CircInteractome database and StarBase database were searched, and it was revealed that miR-382-5p might be a downstream target of circ_0000467 (Figure 3(a)). The data of the luciferase reporter gene experiment showed that miR-382-5p mimics remarkably diminished the luciferase activity of the cells transfected with WT-circ_0000467 plasmid, while the transfection of miR-382-5p had no remarkable effects on the luciferase activity of cells transfected with MUT-circ_0000467 plasmids (Figure 3(b)). Furthermore, RIP and pull-down experiments verified that circ_0000467 specifically bound to miR-382-5p in both SW620 and HT29 cells (Figure 3(c-d)). Additionally, qRT-PCR implied that miR-382-5p was markedly under-expressed in CRC tissues compared within normal tissues adjacent to cancer (Figure 3(e)); miR-382-5p expression was also remarkably down-modulated in CRC cells relative to FHC cells (Figure 3(f)). Besides, miR-382-5p expression was remarkably elevated in both SW620 and HT29 cells after circ_0000467 knockdown (Figure 3(g)). Pearson’s correlation analysis showed a negative link between miR-382-5p and circ_0000467 expressions in CRC tissues (R^2^ = 0.4920, *P* < 0.001, Figure 3(h)). In conclusion, the findings implied that in CRC cells, circ_0000467 adsorbed miR-382-5p and negatively modulated its expression.

**Figure 3.** MiR-382-5p was a downstream target of circ_0000467

a Bioinformatics analysis predicted that the sequence of miR-382-5p matched the sequences of circ_0000467, and WT-circ_0000467 and MUT-circ_0000467 luciferase reporter vectors were constructed.b The miR-382-5p mimics or miR control was co-transfected with WT-circ_0000467 or MUT-circ_0000467, respectively, into HEK293T cells. After 48 h, the luciferase activity of each group of cells was measured.c The complex containing circ_0000467 and miR-382-5p in SW620 and HT29 cells was immunoprecipitated by anti-Ago2, which was confirmed by RIP assay.d RNA pull-down assay was carried out to verify the interactions between circ_0000467 and miR-382-5p.e qRT-PCR was implemented to examine miR-382-5p expression in 69 paired CRC tissues and matched adjacent tissues.f qRT-PCR was employed to examine miR-382-5p expression in CRC cell lines and FHC cells.g MiR-382-5p expression in SW620 and HT29 cells transfected with si-circ_0000467 was detected by qRT-PCR.h Pearson’s correlation analysis was utilized to evaluate the correlations between circ_0000467 expression and miR-382-5p expression in CRC tissues.**P < 0.01, ***P < 0.001, and ‘ns’ indicates that the difference was not statistically significant.

### EN2 was the target of miR-382-5p

StarBase online analysis predicted a complementary binding site between miR-382-5p and the 3'UTR of EN2 (Figure 4(a)). To validate whether miR-382-5p could bind to the 3'UTR of EN2, a dual-luciferase reporter gene experiment was conducted. The findings unearthed that miR-382-5p mimic remarkably weakened the luciferase activity of the cells transfected with WT-EN2 reporter, while it did not markedly alter the luciferase activity of the cells transfected with MUT-EN2 reporter (Figure 4(b)). qRT-PCR and Western blot showed that the up-modulation of miR-382-5p expression remarkably impeded EN2 protein expression in SW620 and HT29 cells (Figure 4(c-d)). Additionally, EN2 was remarkably overexpressed in CRC tissues relative to normal tissues adjacent to cancer (Figure 4(e)). Pearson’s correlation analysis uncovered that miR-382-5p expression was negatively linked to EN2 expression (R^2^ = 0.4702, *P* < 0.001, Figure 4(f)). Western blot experiments also showed that knocking down circ_0000467 inhibited the protein expression of EN2 while co-transfection of miR-382-5p inhibitors partly counteracted the decrease in EN2 expression (Figure 4(g)). Thus, circ_0000467 modulated EN2 expression through regulating miR-382-5p.

**Figure 4.** EN2 was a direct target of miR-382-5p

a Bioinformatics analysis predicted that the sequence of EN2 3’UTR matched the sequence of miR-382-5p, and WT-EN2 and MUT-EN2 luciferase reporter gene vectors were constructed.b The miR-382-5p mimics or miR control was co-transfected with WT-EN2 or MUT-EN2, respectively, into HEK293T cells, and the luciferase activity of each group of cells was measured.c The miR-382-5p mimics were transfected into SW620 and HT29 cells, and the transfection efficiency was detected by qRT-PCR.d Western blot was utilized to detect EN2 protein expression in SW620 and HT29 cells transfected with miR-382-5p mimic.e qRT-PCR was conducted to examine EN2 expression in 69 paired CRC tissues and matched adjacent normal tissues.f Pearson’s correlation analysis was utilized to evaluate the correlations between the expression levels of EN2 and miR-382-5p in CRC tissues.g Western blot was employed to detect EN2 protein expression in SW620 and HT29 cells co-transfected with si-circ_0000467 and miR-382-5p inhibitor.*P < 0.05, **P < 0.01, ***P < 0.001.

### Circ_0000467 enhanced the multiplication, migration, and invasion of CRC cells via miR-382-5p/EN2 axis

To elaborate on whether circ_0000467 affected CRC progression by modulating the miR-382-5p/EN2 axis, ‘compensation tests’ were conducted. CRC cells with circ_0000467 knockdown were co-transfected with pcDNA3.1-EN2. Western blot experiment revealed that circ_0000467 knockdown repressed EN2 protein expression while its protein expression was remarkably augmented after EN2 overexpression plasmids were co-transfected (Figure 5(a)). MTT assay, Transwell experiments, and Western blot showed that circ_0000467 knockdown impeded the multiplication, migration, invasion, and EMT of SW620 and HT29 cells while the suppressing effects of circ_0000467 knockdown on CRC migration, invasion, and EMT process were partially abolished after EN2 overexpression (Figure 5(b-d)). Taken together, it was concluded that circ_0000467 facilitated the multiplication, migration, invasion, and EMT of CRC cells through miR-382-5p/EN2 axis.

**Figure 5.** Circ_0000467 enhanced the multiplication and invasion of CRC cells via miR-382-5p/EN2 axis

a Western blot was employed to detect EN2 protein expression in SW620 and HT29 cells transfected with si-circ_0000467 and pcDNA3.1-EN2.b MTT experiment was conducted to detect the multiplication of SW620 and HT29 cells after the transfection.c Transwell experiment was exploited to detect migration and invasion of SW620 and HT29 cells after the transfection.d Western blot was utilized to detect the EMT markers in SW620 and HT29 cells after the transfection.*P < 0.05, **P < 0.01, and ***P < 0.001.

## Discussion

Accumulating research reports that circRNA dysregulation is strongly linked to CRC development and circRNAs are expected to be novel markers and targets for CRC diagnosis and therapy [9]. In this work, two CRC-related datasets from the GEO database were used to screen differentially expressed circRNAs, the results of which implied that circ_0000467 was remarkably up-modulated in CRC. Circ_0000467 is remarkably overexpressed in gastric cancer tissues, cell lines, and plasma samples of the patients, and circ_0000467 expression is strongly linked to TNM stage [20]. Furthermore, by targeting miR-326-3p and modulating miR-326-3p expression, circ_0000467 facilitates the multiplication and invasion of gastric cancer cells and enhances the number of cells entering G2/M phase [21]. In this work, circ_0000467 was verified to be remarkably overexpressed in CRC tissues and cells, and its expression was associated with tumor size, histological grade, and TNM stage. Additionally, circ_0000467 knockdown markedly suppressed the multiplication, migration, invasion, and EMT of CRC cells, which indicated that circ_0000467 could contribute to CRC progression.

Diverse human miRNAs are dysregulated in cancer [22]. Reportedly, miRNAs can negatively modulate the expression levels of 60% of protein-coding genes, and their dysregulation contributes to cancer development [23,24]. In this work, we predicted and validated that miR-382-5p, which was remarkably down-modulated in CRC tissues and cells, was a direct target of circ_0000467. Reportedly, miR-382-5p modulates the biological behaviors of diverse cancer cells. For instance, in gliomas, miR-382-5p expression is down-modulated and miR-382-5p restrains cancer cell multiplication, migration, invasion, and EMT by targeting the oncogene YBX1 [25]. MiR-382-5p expression is demonstrated to be remarkably down-modulated in both CRC tissues and cell lines [26], which is consistent with our findings. Additionally, the up-modulation of miR-382-5p expression impedes CRC cell multiplication and metastasis by targeting NR2F2 and PD-L1 [27]. Our work also authenticated that circ_0000467 specifically adsorbed miR-382-5p and impeded miR-382-5p expression. The findings imply that circ_0000467 regulates CRC cell multiplication, migration, invasion, and EMT by targeting miR-382-5p.

EN2, a member of the engrailed homeobox family, is evolutionarily conserved and exerts a crucial regulatory effect in regulating the differentiation of mature tissues [19]. EN2 is an essential transcription factor that precisely modulates cell differentiation by specifically activating downstream genes [28]. Moreover, EN2 exerts a carcinogenic or tumor-suppressive role in different cancers. For instance, in renal clear cell carcinoma and non-small cell lung cancer (NSCLC), EN2 expression is down-modulated and negatively linked to the clinicopathological stage [29,30]. EN2 overexpression impedes the multiplication and metastasis of NSCLC cells [30]. EN2 is under-expressed in gliomas, and elevated EN2 expression restrains cell multiplication, enhances tumor sensitivity to temozolomide, and blocks tumor cell invasion by repressing MMP9 expression [31]. Conversely, in ovarian cancer, high EN2 expression predicts the adverse prognosis of the patients [18]. In prostate cancer, EN2 facilitates cell cycle and multiplication of cancer cells through regulating PI3K/AKT pathway [32]. Importantly, EN2 works as an oncogene in CRC, and EN2 overexpression is remarkably associated with the unfavorable prognosis of the patients; furthermore, *in vivo* experiments show that EN2 enhances CRC multiplication and migration by modulating CCL20 expression [19]. In this work, EN2 was revealed to be a direct downstream target of miR-382-5p, and positively regulated by circ_0000467. Compensation experiment revealed that EN2 overexpression partially counteracted the suppressing effects of circ_0000467 depletion on CRC cell multiplication, migration, invasion, and EMT. These data imply the circ_0000467 exerts its oncogenic functions in CRC via regulating miR-382-5p and EN2.

## Conclusion

In summary, this work substantiates that circ_0000467 expression is remarkably up-modulated in CRC tissues and circ_0000467 overexpression is linked to unfavorable pathological characteristics in CRC patients. We confirm that circ_0000467 facilitates CRC development through the miR-382-5p/EN2 pathway (Figure 6). The findings of this work imply that circ_0000467 may be a new therapeutic target for CRC patients.

**Figure 6.** Graphic abstract: Depletion of circ_0000467 suppressed the malignant phenotypes of CRC cells via modulating the expression levels of miR-382-5p and EN2

## Data Availability

The data used to support the findings of this study are available from the corresponding author upon request.

## Highlights

1. Circ_0000467 is highly expressed in CRC.
2. Circ_0000467 affects the multiplication, migration, invasion, and EMT processes of CRC cells.
3. Circ_0000467 functions as a sponge of miR-382-5p in CRC cells.

EN2 is a target of miR-382-5p.
